# Analysis on the Expression and Prognostic Value of LncRNA FAF in Patients with Coronary Heart Disease

This article has been retracted.

**DOI:** 10.1155/2020/9471329

**Published:** 2020-11-02

**Authors:** Hai Xu, Xiwen Zhang, Kun Yu, Gang Zhang, Yafei Shi, Yicheng Jiang

**Affiliations:** Department of Cardiology, The Affiliated Huaian No. 1 People's Hospital of Nanjing Medical University, Huai'an 223000, China

## Abstract

**Objective:**

To investigate the expression and prognostic value of LncRNA FAF in patients with coronary heart disease. *Patients and Methods*. 97 patients with coronary heart disease who came to our hospital were selected as the research group (RG), and 97 healthy people who came to our hospital for physical examination during the same period were selected as the control group (CG). The serum LncRNA FAF, plasma homocysteine (HCY), lipoprotein A (Lp-a), serum tumor necrosis factor *α* (TNF-*α*), and high-sensitivity C-reactive protein (hsCRP) in the two groups of patients were detected, and their correlations were analyzed. Then, the predictive value and risk factors of FAF for poor prognosis of patients with coronary heart disease were analyzed.

**Results:**

The expression of LncRNA FAF in the serum of patients in the RG was significantly lower than that in the CG, and the expressions of HCY, Lp-a, TNF-*α*, and hsCRP were significantly higher than those in the CG (*p* <0.05). The AUC of FAF in the diagnosis of coronary heart disease was more than 0.9. FAF was negatively correlated with the coronary lesion vessels, HCY, Lp-a, TNF-*α*, and hsCRP expressions in patients with coronary heart disease (*p* < 0.05). The ROC of FAF for predicting poor prognosis in patients with coronary heart disease was greater than 0.9. Low expression of FAF; high expressions of HCY, Lp-a, and hsCRP; and increase of coronary lesion vessels were independent risk factors for poor prognosis in patients with coronary heart disease.

**Conclusions:**

LncRNA FAF was lowly expressed in the serum of patients with coronary heart disease, and it was of high value in the diagnosis and prediction of poor prognosis of coronary heart disease. It was also an independent risk factor for poor prognosis of patients with coronary heart disease and may be a potential target for diagnosis and treatment of coronary heart disease.

## 1. Introduction

In recent years, with the changes of social environment and the improvement of living standards, the incidence rate of cardiovascular diseases is getting higher. Coronary heart disease is one of the most common cardiovascular diseases, and acute myocardial infarction caused by coronary heart disease is also one of the main causes of disability or death in patients with cardiovascular diseases, which poses a serious threat to human health [1, 2]. At present, coronary heart disease patients are mainly diagnosed and treated by cardiovascular intervention technology [3]. Although great progress has been made in the diagnosis and treatment of coronary heart disease with the development of medical technology, there are still a large number of patients with coronary heart disease who cannot be diagnosed and evaluated in time, resulting in patients who cannot be treated in time in sudden situations such as myocardial infarction [4, 5]. Therefore, how to timely and effectively diagnose and treat patients with coronary heart disease is also one of the problems that need to be solved urgently in clinical practice.

In recent years, with the development of molecular biology, the application of molecular targeted diagnosis and treatment technology in cardiovascular diseases is becoming more and more extensive, take long noncoding RNA ANRIL, for example [6]. Long noncoding RNA (LncRNA) is a noncoding RNA with a length of more than 200 nt. In the past, LncRNA has been reported to play an important role in the occurrence of many diseases, including cardiovascular diseases [7]. For example, previous studies [8] found that LncRNA NEAT1 can inhibit vascular endothelial cell injury induced by oxidative stress by activating miR-181d-5p/CDKN3 axis. LncRNA FAF is the latest LncRNA related to cardiovascular diseases [9]. Recent studies [9] have suggested that it can inhibit apoptosis of ischemic and hypoxic myocardial cells together with the upregulation of fibroblast growth factor (FGF9), but its clinical value in coronary heart disease has not been elaborated. FGF9 is a factor that has been proved to play an important regulatory role in myocardial infarction, and it is believed to play an important regulatory role in coronary artery vascular development [10], so we speculated whether LncRNA FAF also plays an important role in the occurrence of coronary heart disease. However, at present, no studies were analyzed on the expression and clinical value of LncRNA FAF in patients with coronary heart disease.

In order to carry out more analysis of LncRNA FAF on the basis of previous scholars, we analyzed the expression of LncRNA FAF in the serum of patients with coronary heart disease and its value in the diagnosis and prognosis of coronary heart disease, so as to improve more clinical data for the diagnosis and treatment of coronary heart disease.

## 2. Materials and Methods

From January 2016 to May 2018, 97 patients with coronary heart disease who visited our hospital were selected as the RG, including 52 male and 45 female, with an average age of (52.34 ± 6.48) years old. 97 healthy people who came to our hospital for physical examination during the same period were selected as the CG, including 54 male and 43 female, with an average age of (53.04 ± 6.52) years old. All patients and their families agreed to participate in the experiment, which has been approved by the hospital ethics committee. (No. K(S)16-14).

The inclusion criteria are patients diagnosed as having coronary heart disease by coronary artery CT angiography.

The exclusion criteria are patients with serious blood system diseases; patients with other malignant tumor diseases; patients with severe immune system diseases; and patients with severe liver and kidney dysfunction.

### 2.1. Detection of FAF Expression by qRT-PCR

5 mL of venous blood was taken from all subjects on an empty stomach and then centrifuged at a temperature of 4°C for 10 min at a speed of 1500 × g. After centrifugation, a supernatant was taken for detection. TRIzol was added to the serum to extract total RNA. The purity, concentration, and integrity of total RNA were detected by a UV spectrophotometer and agarose gel electrophoresis. cDNA reverse transcription was performed according to the kit instructions (TransGen Biotech, Beijing, China), and FAF detection was performed according to the kit instructions. The FAF amplification system was as follows: cDNA 1 *μ*L, upstream and downstream primers each 0.4 *μ*L, 2X SYBR Green mixture 10 *μ*L, and Passive Reference Dye (50X) 0.4 *μ*L. In the end, ddH_2_O was added to complete to 20 *μ*L. Amplification conditions were as follows: PCR reaction conditions: predegeneration at 95°C for 30 s, degeneration at 95°C for 5 s, anneal and extension at 60°C for 15 s, then followed by a total of 40 cycles. GAPDH was used as an internal parameter. Primer sequences are shown in Table 1. The experiment was repeated three times.

### 2.2. Detection of Other Related Indexes

We detected cardiovascular disease-related factors and related inflammatory factors in the serum of patients in the RG, including plasma homocysteine (HCY), lipoprotein A (Lp-a), serum tumor necrosis factor *α* (TNF-*α*), and high-sensitivity C-reactive protein (hsCRP). PAF, ET-1 and TNF-*α* (Shanghai Meilian Biotechnology Co., Ltd.) were detected by ELISA. The operation was strictly in accordance with the kit instructions. Immunofluorescence quantitative was used to detect the expression of hsCRP (Boditech Med Inc.).

### 2.3. Statistical Methods

In this study, SPSS20.0 was used for statistical analysis of experimental data. The counting data were tested by the chi-squared test. The measurement data were expressed as mean number ± standard deviation. *t*-test was used for comparison between the two groups. The paired *t*-test was used for the comparison before and after treatment. Pearson correlation was used for correlation analysis. Logistic regression model was used to analyze the risk factors of adverse cardiovascular events. GraphPad Prism 6 was used to draw the images in this experiment. There was a statistical difference with *p* < 0.05.

## 3. Results

### 3.1. Baseline Data

There was no significant difference in gender, age, and BMI between the two groups (*p* > 0.05), but there was significant difference in the number of hypertension (*p* < 0.05). More details are shown in Table 2.

### 3.2. Comparison of Serum FAF Expression between the Two Groups of Subjects

The FAF expression of patients in the RG was 0.63 ± 0.12, significantly lower than that in the CG (0.91 ± 0.15), and the difference was statistically significant (*p* < 0.05). We analyzed the FAF in patients in the RG, and the results indicated that the expression of serum FAF in patients with multivessel coronary artery disease (0.45 ± 0.08) was significantly lower than that in patients with double-vessel (0.61 ± 0.08) and single-vessel disease (0.73 ± 0.08), and the expression of serum FAF in patients with double-vessel disease was significantly lower than that in patients with single-vessel disease, and the differences were statistically significant (*p* < 0.05). More details are shown in Figure 1.

### 3.3. Expression of HCY, Lp-a, TNF-*α*, and hsCRP in Serum of Subjects in the Two Groups

The expressions of HCY (24.42 ± 5.31) umol/L, Lp-a (214.15 ± 26.47) mmol/L, TNF-*α* (66.27 ± 7.31) pg/mL, and hsCRP (8.49 ± 1.31) mg/L in the RG of patients were significantly higher than those of HCY (8.26 ± 1.67) umol/L, Lp-a (91.33 ± 14.62) mmol/L, TNF-*α* (32.16 ± 2.84) pg/mL, and hsCRP (4.02 ± 0.83) mg/L in the CG. The difference was statistically significant (*p* < 0.05). More details are shown in Figure 2.

### 3.4. Diagnostic Value and Correlation Analysis of FAF for Coronary Heart Disease

ROC curve analysis indicated that the AUC of FAF in the diagnosis of coronary heart disease was 0.935, which had a high diagnostic value. Moreover, there was a negative correlation between FAF and coronary lesion vessels and the expression of HCY, Lp-a, TNF-*α*, and hsCRP in serum of patients with coronary heart disease (*p* < 0.05). More details are shown in Figure 3.

### 3.5. The Predictive Value of FAF for Poor Prognosis in Patients with Coronary Heart Disease

All patients with coronary heart disease were followed up for one year. Patients were divided into a MACE group (40 cases) and non-MACE group (57 cases) according to the occurrence of adverse cardiac events (MACE) during the follow-up period. After comparing the serum FAF in the two groups of patients, it was found that the serum FAF of patients in the MACE group was significantly lower than that in the non-MACE group (*p* < 0.05). ROC analysis indicated that the AUC of FAF for predicting poor prognosis of patients with coronary heart disease was 0.916, which had high predictive value. More details are shown in Figure 4.

### 3.6. Univariate Analysis of Poor Prognosis in Patients with Coronary Heart Disease

After univariate analysis of patients in the MACE group and non-MACE group, it was found that there were no significant differences in gender, age, drinking, and other aspects between the two groups (*p* > 0.05), and there were significant differences in FAF, HCY, Lp-a, hsCRP, and lesion vessels (*p* < 0.05). More details are shown in Table 3.

### 3.7. Multivariate Analysis of Poor Prognosis in Patients with Coronary Heart Disease

We included FAF, HCY, Lp-a, hsCRP, and lesion vessels for analysis and listed them as dependent variables for assignment (Table 4). MACE or not was taken as the dependent variable. The logistic regression model was used for multivariate analysis. The results indicated that FAF, HCY, Lp-a, hsCRP, and lesion vessels were independent risk factors for poor prognosis of coronary heart disease patients (Table 5).

## 4. Discussion

In recent years, with the development of sequencing technology, LncRNA has also been discussed as a key research direction in the research of cardiovascular diseases. Many mechanisms of LncRNA in diseases have been extensively studied and elaborated [11, 12]. Coronary artery disease is one of the major types of cardiovascular diseases. Due to the limited treatment methods and the side effects caused by long-term drug use, there are still great challenges in the early diagnosis and treatment of coronary heart disease [13, 14]. LncRNA is a potential diagnosis and treatment target for coronary heart disease in the future, and there are also many related researches. For example, previous studies [15] indicated that the specificity of plasma LncRNA marker for diagnosis of coronary heart disease can reach more than 90%.

This study was designed to discuss the expression of LncRNA FAF in the serum of patients with coronary heart disease and its related clinical significance. FAF belongs to LncRNA which is found to be abnormally expressed in cardiovascular diseases. In the past, many researches have been conducted on the mechanism of LncRNA in coronary artery diseases. For example, research [16] concluded that LncRNA HOTTIP can promote the proliferation and migration of vascular endothelial cells by activating the Wnt/*β*-catenin pathway. Other studies [17] have found that the level of LncRNA H19 in plasma was related to the risk of coronary artery disease. However, there are few related studies on FAF. Previous studies [9] claimed that LncRNA FAF and FGF9 were located on the same chromosome and can be combined by reverse complementation. In our study, we first found that FAF was low expressed in the serum of patients with coronary heart disease and found that it had high value in the diagnosis of coronary heart disease and the prediction of poor prognosis of coronary heart disease. In the past research [18], it was said that FGF9 can improve the systolic function of the heart by reducing interstitial fibrosis, thus reducing the mortality rate of heart failure. A study [19] pointed out that LncRNA FAF can inhibit cardiac fibrosis by targeting FGF9. In this study, it was found that FAF was lowly expressed in the process of myocardial fibrosis, which is similar to our conclusion.

Then, in order to further analyze the relationship between FAF and coronary heart disease, we first detected the expressions of HCY, Lp-a, TNF-*α*, and hsCRP in the serum of patients with coronary heart disease. The results indicated that the expressions of HCY, Lp-a, TNF-*α*, and hsCRP in the serum of patients with coronary heart disease were significantly higher than those in the CG. HCY is a sulfur amino acid in the metabolic process of human cells, and its content is generally lower in the human body [20]. Previous studies [21] pointed out that the higher the level of HCY, the greater the risk of cardiovascular diseases. Lp-a, as a protein complex synthesized in the liver, can prevent blood clot dissolution in blood by combining with fibrin, which is the main cause of atherosclerosis [22]. TNF-*α* and hsCRP both belong to inflammatory factors. In coronary heart disease, hsCRP is more representative as one of inflammatory markers, which can directly induce monocytes to aggregate into atherosclerotic plaques, thus causing vascular endothelial dysfunction [23]. The increase of the serum hsCRP level in patients with coronary heart disease often represents the more serious myocardial injury in patients [24]. Through correlation analysis, we found that FAF was negatively correlated with the expressions of HCY, Lp-a, TNF-*α*, and hsCRP in the serum of patients with coronary heart disease, which indicated that FAF may be closely related to the formation of coronary heart disease and myocardial injury, but the specific regulatory relationship between FAF and myocardial injury is still unclear. In the past, there are relatively many studies on other LncRNA in coronary heart disease. For example, LncRNA-LET can reduce hypoxia-induced myocardial cell damage by regulating miR-138 [25]. There are also studies [26] that pointed out that LncRNA BANCR may be used as a biomarker for the screening and prevention of coronary heart disease. However, the research on FAF in coronary heart disease is still at a relatively blank stage. Then, in order to further enrich our data, we analyzed the risk factors for poor prognosis of patients with coronary heart disease by logistic multiple regression. The results indicated that low expression of FAF and high expression of HCY, Lp-a, hsCRP, and multivessel coronary artery disease were independent risk factors for poor prognosis of patients with coronary heart disease. In the past, previous studies clearly pointed out that elevated HCY, Lp-a, and hsCRP were independent risk factors for coronary heart disease [27, 28], which is similar to our conclusion. The increase of coronary lesion vessels also represented that the patient's condition was more serious, which may also be one of the causes for the occurrence of MACE in patients [29]. However, this is the first time that we have found that the low expression of FAF is an independent risk factor for poor prognosis of patients with coronary heart disease, but more studies are needed to prove it in the future.

There are still some deficiencies in this study. For example, we have not explored the role of FAF in coronary heart disease from basic experiments. Secondly, due to the lack of relevant studies, a large number of experiments are still needed to demonstrate our research.

## 5. Conclusions

To sum up, LncRNA FAF was lowly expressed in the serum of patients with coronary heart disease, and it was of high value in the diagnosis and prediction of poor prognosis of coronary heart disease. It was also an independent risk factor for poor prognosis of patients with coronary heart disease and may be a potential target for the diagnosis and treatment of coronary heart disease.

## Figures and Tables

**Figure 1:** Comparison of serum FAF expression between the two groups of subjects. (a) The expression of FAF in the RG was significantly lower than that in the CG. (b) The expression of serum FAF in patients with multivessel coronary artery disease was significantly lower than that in patients with double-vessel and single-vessel disease, and the expression of serum FAF in patients with double-vessel disease was significantly lower than that in patients with single-vessel disease. ∗ indicates *p* < 0.05.

**Figure 2:** Expression of HCY, Lp-a, TNF-*α*, and hsCRP in serum of subjects in the two groups. (a) HCY expression in the RG was significantly higher than that in the CG. (b) Lp-a expression in the RG was significantly higher than that in the CG. (c) TNF-*α* expression in the RG was significantly higher than that in the CG. (d) hsCRP expression in the RG was significantly higher than that in the CG. ∗ indicates *p* < 0.05.

**Figure 3:** Diagnostic value and correlation analysis of FAF for coronary heart disease. (a) ROC analysis of FAF in the diagnosis of coronary heart disease. (b) There was a negative correlation between FAF and coronary lesion vessels in patients with coronary heart disease (*r* = −0.881, *p* < 0.001). (c) The FAF and PAF expressions were negatively correlated (*r* = −0.728, *p* < 0.001). (d) FAF and ET-1 expressions were negatively correlated (*r* = 0 − 704, *p* < 0.001). (e) FAF and TNF-*α* expressions were negatively correlated (*r* = −0.674, *p* < 0.05). (f) FAF and hsCRP expressions were negatively correlated (*r* = −0.664, *p* < 0.05).

**Figure 4:** The predictive value of FAF for poor prognosis of patients with coronary heart disease: (a) low expression of FAF in serum of patients with poor prognosis of coronary heart disease; (b) the predictive value of FAF for poor prognosis of patients with coronary heart disease. ∗ indicates *p* < 0.05.

**Table 1:** Primer sequence.

Factors	Upstream primers	Downstream primers
FAF	5′-CGCTAAAGGCACAGGGTCAG-3′	5′-CACCAACCTTTCCCTTCCAGTC-3′
GAPDH	5′-GGCACAGTCAAGGCTGAGAATG-3′	5′-ATGGTGGTGAAGACGCCAGTA-3′

**Table 2:** Baseline data.

Factors	RG	CG	*t*/*χ*^2^	*p*
	*n* = 97	*n* = 97		
Gender			0.083	0.773
Male	52 (53.61)	54 (55.67)		
Female	45 (46.39)	43 (44.33)		
Age/years old	52.34 ± 6.48	53.04 ± 6.52	0.750	0.454
BMI (kg/m^2^)	23.54 ± 2.16	23.66 ± 2.21	0.382	0.703
Types			—	—
Myocardial infarction	42 (43.30)	—		
Nonmyocardial infarction	55 (56.70)	—		
Count of coronary artery stenosis			—	—
Single vessel	31 (31.96)	—		
Double vessel	35 (36.08)	—		
Multiple vessels	32 (32.99)	—		
Drinking history			0.083	0.774
Yes	52 (53.61)	50 (51.55)		
No	45 (46.39)	47 (48.45)		
Smoking history			0.021	0.885
Yes	43 (44.33)	44 (45.36)		
No	54 (55.67)	53 (54.64)		
Hypertension			8.269	0.004
Yes	61 (62.89)	41 (42.27)		
No	36 (37.11)	56 (57.73)		

**Table 3:** Univariate analysis of poor prognosis in patients with coronary heart disease.

Factors	MACE group	Non-MACE group	*t*/*χ*^2^	*p*
	*n* = 40	*n* = 57		
Gender (*n* (%))			0.053	0.818
Male	22 (55.00)	30 (52.63)		
Female	18 (45.00)	27 (47.37)		
Age/years old	52.26 ± 6.35	52.44 ± 6.51	0.135	0.893
BMI (kg/m^2^)	23.49 ± 2.22	23.58 ± 2.18	0.199	0.843
Lesion vessels			7.406	0.025
Single vessel	10 (25.00)	21 (36.84)		
Double vessel	11 (27.50)	26 (45.61)		
Multiple vessels	19 (47.50)	13 (22.81)		
FAF	0.43 ± 0.09	0.71 ± 0.13	11.78	<0.001
HCY (*μ*mol/L)	26.31 ± 4.26	20.09 ± 3.81	7.537	<0.001
Lp-a (mmol/L)	228.45 ± 18.31	202.66 ± 15.73	7.426	<0.001
TNF-*α* (pg/mL)	67.26 ± 7.02	66.05 ± 7.11	0.829	0.409
hsCRP (mg/L)	9.63 ± 1.02	7.83 ± 1.06	8.361	<0.001

**Table 4:** Assignment table.

Factors	Assignment
Lesion vessels	Single vessel, double vessel = 1, multiple vessels = 2
FAF	Data belonged to continuous variables and was analyzed with original data
HCY	Data belonged to continuous variables and was analyzed with original data
Lp-a	Data belonged to continuous variables and was analyzed with original data
hsCRP	Data belonged to continuous variables and was analyzed with original data

**Table 5:** Multivariate analysis of poor prognosis in patients with coronary heart disease.

Factor	*β*	S.E	Wald	OR	95% CI	*p*
Lesion vessels	0.459	0.211	4.662	1.631	1.042-2.419	0.028
FAF	0.919	0.187	25.073	2.521	1.751-3.611	<0.001
HCY	0.437	0.141	9.154	1.537	1.169-2.029	0.002
Lp-a	1.085	0.467	5.273	2.991	1.176-7.521	0.023
hsCRP	0.982	0.368	7.009	2.693	1.288-5.563	0.007

## Data Availability

The data can be unconditionally disclosed.
